# Application Analysis of Multidisciplinary Diagnosis and Treatment Nursing Mode Based on Doctor-Nurse-Integration for Stroke Patients Undergoing Emergency Intervention Surgery

This article has been retracted.

**DOI:** 10.1155/2022/6299676

**Published:** 2022-11-11

**Authors:** Hai Zhong, Aiqun Liang, Huanhuan Luo, Xiaolong Hu, Shengxiang Xu, Ziming Zheng, Xiaoping Zhu

**Affiliations:** ^1^Wuhan University School of Nursing, Wuhan, Hubei 430071, China; ^2^Intervention Operating Room, Zhongshan City People's Hospital, Zhongshan, Guangdong 528403, China

## Abstract

**Purpose:**

To analyze the application value of multidisciplinary diagnosis and treatment (MDT) nursing mode based on doctor-nurse-integration for stroke patients undergoing emergency intervention surgery.

**Methods:**

In this study, a historical comparative study method was adopted. 118 stroke patients and medical staff (9 doctors and 11 nurses) who met the diagnosis and inclusion criteria of emergency intervention surgery admitted from July 2021 to February 2022 were treated clinically according to the traditional medical care mode (TMC group), 87 stroke patients and medical staff (9 doctors and 11 nurses) who met the diagnosis and inclusion criteria of emergency intervention surgery admitted from February 2022 to June 2022 were treated and cared according to the MDT nursing mode based on medical integration (MDT group). Comparison of perioperative time indicators, postoperative outcome indicators, treatment compliance, secondary complications and visit satisfaction between the two groups of patients, and comparison of cooperation satisfaction between the two groups of medical staff.

**Results:**

The MDT group had shorter onset—emergency physician's reception time, arrival at CT room—completion time of CT/MR, notify intervention chamber—arrival time at catheter chamber, admission—femoral artery puncture time, admission—first vessel recanalization time, mean postural restraint time than the TMC group (*P* < 0.05). The postoperative mortality rate in the MDT group (5.75%) was comparable to that in the TMC group (8.47%) (*P* > 0.05); the postoperative disability rate in the MDT group (28.74%) was less than that in the TMC group (45.76%) (*P* < 0.05); the NIHSS score in the MDT group was lower than that in the TMC group, and the FMA score and BI score were both higher than those in the TMC group (*P* < 0.05). The MDT group had higher treatment compliance than the TMC group, fewer secondary complications than the TMC group, and higher patient visit satisfaction and medical staff cooperation satisfaction than the TMC group (*P* < 0.05).

**Conclusion:**

The implementation of the MDT nursing mode based on the doctor-nurse-integration for stroke patients undergoing emergency intervention surgery can improve the work efficiency of rescuing patients, improve the clinical treatment outcome of patients, and improve the satisfaction of doctors, nurses, and patients.

## 1. Introduction

The incidence of stroke in China is currently on the rise, with more than half of those who survive showing varying degrees of loss of ability to perform daily activities. A study by Barthels and Das [1] showed that the most significant disease causing long-term disability in Western countries is stroke and that the functional impairment of stroke sequelae severely reduces the quality of life of patients. Intravenous thrombolysis is the standard of care for acute ischemic stroke (AIS) [2]. Studies [3] have shown that mechanical thrombectomy has become the mainstay of treatment for large vessel occlusion in AIS and is effective in reducing the mortality and disability rates in AIS patients. However, due to factors such as the short time window for treatment, only a small number of patients are able to receive timely and effective treatment. Therefore, an efficient stroke care system that works within a limited time window is key to improving the efficiency of care [4]. Multidisciplinary diagnosis and treatment (MDT) refers to the diagnosis and treatment mode in which two or more disciplines in the clinic can put forward the best treatment plan for a clinical disease through multidisciplinary expert discussion [5]. In recent years, MDT has become an important diagnosis and treatment mode in the international medical field, promoting multidisciplinary cooperation and improving diagnosis and treatment efficiency and success rate [6]. In addition, the cooperative behavior of doctors and nurses is also an important factor that directly affects the medical quality, medical relations, patient health solutions, and patient satisfaction [7, 8]. The clinical nursing mode of doctor-nurse-integration requires nurses to integrate the idea of doctor and patient participation in clinical nursing work such as nursing procedures and health education, through benign communication and good cooperation, the doctors and nurses jointly formulate diagnosis and treatment plans to realize the complementarity of specialized knowledge and professional skills between the doctors and nurses, patients and caregivers receive consistent and standardized scientific rehabilitation guidance and help from different aspects, providing a good treatment and nursing environment for patients. The purpose of this study is to explore the application value of MDT nursing model based on doctor-nurse-integration in stroke patients undergoing emergency intervention surgery.

## 2. Materials and Methods

### 2.1. Research Object

In this study, a historical comparative study method was adopted. 118 stroke patients and medical staff (9 doctors and 11 nurses) who met the diagnosis and inclusion criteria of emergency intervention surgery admitted from July 2021 to February 2022 were treated clinically according to the traditional medical care mode (TMC group), 87 stroke patients and medical staff (9 doctors and 11 nurses) who met the diagnosis and inclusion criteria of emergency intervention surgery admitted from February 2022 to June 2022 were treated and cared according to the MDT nursing mode based on medical integration (MDT group). Inclusion criteria: those who met the American Heart Association [9] diagnostic criteria for AIS and confirmed the diagnosis in combination with CT or MRI; those who had a complete medical history; those who were aware of the study and signed to confirm; those who had their first episode; those who were within 24 h of onset to admission; and those over 18 years of age. Exclusion criteria: those with recurrent stroke; those with severe circulatory, digestive, respiratory, endocrine system diseases, or malignant tumors that seriously affect the quality of life; those with severe aphasia, cognitive impairment, dementia, and psychosis, unable to cooperate with the investigator; those with a clear history of bleeding tendencies or contraindications to endovascular treatment, those who were pregnant, and coagulation disorders; those who refused to agree to sign the interventional procedure consent form; those who withdrew themselves from the included cases and did not complete treatment. Statistical differences in Table 1 for baseline information of both groups were analysed, *P* > 0.05, comparable.

## 3. Care Methods

### 3.1. TMC Group: Clinical Treatment and Care According to the Traditional Medical Care Work Pattern

(1) Initial screening of ischemic stroke patients, emergency triage nurses quickly identified stroke patients based on their condition within 10 minutes, and a greenway would be activated for suspected stroke patients to notify the neurology resident and escort the patient to the resuscitation unit. (2) Those eligible for initial screening into the greenway, with a diagnosis considered to be AIS, onset <24 h and age 18 years or older. (3) After completing the preliminary screening preparation and entering the greenway, the nurses in the rescue room quickly established venous channels, collected test samples, inquired about the medical history, judged the condition, and improved the preparations before ECG and CT examination. The neurology resident arrived for consultation within 15 minutes of notification, and completed the CT examination within 25 minutes, the CT examination report was issued within 45 minutes. (4) Within 60 minutes, the resuscitation room nurse cooperated with thrombolytic therapy in the CT room. If the CT result showed that the large vessel was occluded, it was immediately sent to the interventional catheterization chamber for revascularization. (5) Preparation for interventional embolectomy, the emergency nurse and the interventional catheterization chamber nurse conducted a handover according to the routine procedure, three checks-seven pairs-one turn to look at the skin condition of each area, and the surgical nurse performed various checks and assessments on the patient, including the consent form for the procedure, the time of reception, the medication, the skin condition, the pipeline condition, and the level of cooperation. (6) Preparation for entry into the interventional suite, patients were allowed to lie flat on the DSA machine bed and placed in a good position, those undergoing head radiography were fixed with special pillows. The ECG monitoring instrument was connected, various pipelines and corresponding rescue instruments were fixed, and the venous indwelling needle was unblocked. (7) Communicate and respond with neurology physician after operation.

### 3.2. MDT Group: Clinical Treatment and Care According to the MDT Nursing Mode Based on Doctor-Nurse-Integration

(1) Formation of an stroke doctor-nurse-integration MDT team: The doctor-nurse-integration clinical care model was adopted, construction of specialized medical care unit for stroke, which provided treatment, nursing, rehabilitation, health education, and other medical and nursing services for stroke patients in the form of doctor-nurse-integration team and multidisciplinary team. The core team consisted of 2 experienced neurologists, 1 emergency room physician, 2 imaging physicians, 1 laboratory physician, 1 anesthetist, 1 rehabilitation physician, 2 nurse-in-charge, 1 technician each in the interventional theater, and 9 trained specialist stroke nurses. All graduated at least 5 years ago and had been in their specialty for at least 3 years, with a relatively fixed mix and grouping of doctors and nurses according to their respective titles and ranks. (2) Development of job responsibilities for members within the group: The director of neurology and the head nurse of the interventional operation room served as the group leader and deputy group leader, respectively, the chief resident physician of neurology coordinated the organization and implementation in a unified manner, and jointly formed the core management team of stroke doctor-nurse-integration MDT team. The 3 persons were responsible for developing the workflow of the team and arranging for the relevant physicians in charge of their specialty to actively cooperate and participate in stroke treatment; a monthly multidisciplinary case discussion was conducted to optimize the treatment process; were responsible for systematic training of the professional staff to keep abreast of the development of stroke treatment at home and abroad. The other members of the team, under the decision and guidance of the core team, followed the coordination and arrangements, were responsible for the implementation and dissemination of information involving the treatment of their specialty, and dynamically reported on the stage of the process and the status of the patient's condition. (3) Integration work of the team: ①According to the guideline [10] and the operation system of our hospital, the neurologist developed the flow chart of multidepartment linkage treatment for AIS patients with emergency interventional treatment (Figure 1). ②A flow chart for rapid identification of stroke patients was prominently displayed in the emergency department, and doctors and nurses used a scale [11] to quickly identify and activate the greenway. ③Measures for greenway access: Patients eligible for greenway access were given priority treatment by special arrangement according to the principle of saving first and paying later. A stroke unit was set up in the resuscitation room and doctors chose the greenway entrance in the doctor's consultation system for medical prescriptions, test orders and checklists, etc. Test specimen tubes were marked with green ribbons and placed on the conveyor belt to reach the testing department directly and the testing department was informed by telephone. (4) Clinical implementation: ①Establishment of an hospital stroke emergency greenway App: Relevant department personnel or doctors on duty push the information of patients treated by greenway on the App interface, the content included basic information, contact information, creation time, push time, data of specific time period, basic vital signs (blood pressure, body mass, blood collection time, rapid blood glucose results, electrocardiogram, NIHSS score, etc.), and treatment information. ②Shorten the treatment time: the consent for interventional operation was signed together with the informed consent for CT examination and thrombolysis, and the intervention room was started in advance. The neurologist and the emergency room nurse nurse prepared the intravenous thrombolysis kit and resuscitation drugs and sent the patient to the CT room. If a large vessel occlusion was found during the CT examination, the patient did not need to wait for the imaging report, and intravenous thrombolysis was performed immediately if it was within the thrombolysis time window, otherwise the patient was sent directly to the interventional catheterization laboratory for revascularization. ③Simplify shift handover: Emergency nurses and nerve physician confirmed the surgical consent form and picked up the patient straight into the interventional operating room, other patient information can be viewed on the App after entering the surgery, shortening shift handover time. ④Emergency protocol for stroke surgery was established to train nurses in emergency response and to improve interventional techniques of neurologists. The nurses in the operating room should be trained and assessed on rescue skills every month to ensure that everyone was proficient in nerve interventional operation. The surgical materials and drugs were backed up and put in special use, and there was a special logo for the stroke greenway, so as to be in emergency at any time; interventional operation room nurses achieved the intervention room within 20 minutes after receiving the call, so as to quickly cooperate with doctors for surgery and achieve the purpose of treatment. ⑤Doctors and nurses worked together to formulate the rescue process and nursing focus of emergency intervention surgery for stroke, fully evaluate the patient's consciousness state, activity level, cooperation degree, upper limb muscle strength level, etc., and then evaluate the necessity of physical restraint of the patient, if restraint was needed, informed consent was obtained, the restraint level was judged, and the restraint was carried out safely and effectively to reduce the patients' anxiety, uncontrolled consciousness, and noncooperation during the operation. Restraint and fixation positions: head, upper limbs, lower limbs, and pipeline (infusion tube, urinary tube), it was ensured that various monitoring cables were firmly connected to avoid falling off and affecting the observation of the disease and the operation of doctors. ⑥Complication management: in case of complications such as technical or hyperperfusion hemorrhage and massive cerebral infarction during and after surgery, the condition and imaging information would be pushed in the app in time and neurologist would be contacted to follow up the treatment and play the role of MDT team.

### 3.3. Observation Index

#### 3.3.1. Perioperative Time Indicators

The main categories included onset—emergency physician's reception time, arrival at CT room—completion time of CT/MR, notify intervention chamber—arrival time at catheter chamber, admission—femoral artery puncture time, admission—first vessel recanalization time, mean postural restraint time.

#### 3.3.2. Postoperative Outcome Indicators

The main components were mortality rate, disability rate, National Institute of Health stroke scale (NIHSS) score, Fugl-Meyer assessment (FMA) score, and Barthel index (BI) score.

#### 3.3.3. Treatment Compliance

Compliance was assessed on the basis of the patient's treatment performance and was graded into three levels: excellent (active and cooperative with nursing operations), good (able to cooperate with nursing operations when supervised by the nurse), and inferior (presence of significant resistance or refusal behavior).

#### 3.3.4. Secondary Complications

The occurrence of postoperative complications such as shoulder subluxation, shoulder hand syndrome, foot drop, inversion of the foot, joint contracture, and urinary tract infection was documented.

#### 3.3.5. Satisfaction

This included 2 levels of patient visit satisfaction and medical staff cooperation satisfaction. Both were designed by the MDT team itself.

### 3.4. Statistical Methods

SPSS 22.0 software was applied. For statistical data (%), *χ*^2^ test was used for comparison between the groups. For measurement data (*M* ± SD), *t*-test was used for comparison between the groups. *P* < 0.05 was considered a statistically significant difference.

## 4. Results

### 4.1. Perioperative Time Indicators

The MDT group had shorter onset—emergency physician's reception time, arrival at CT room—completion time of CT/MR, notify intervention chamber—arrival time at catheter chamber, admission—femoral artery puncture time, admission—first vessel recanalization time, mean postural restraint time than the TMC group, all with statistically significant differences (*P* < 0.05) (Figure 2).

### 4.2. Postoperative Outcome Indicators

The postoperative mortality rate in the MDT group (5.75%) was comparable to that in the TMC group (8.47%), and the difference was not statistically significant (*P* > 0.05); the postoperative disability rate in the MDT group (28.74%) was less than that in the TMC group (45.76%), and the difference was statistically significant (*P* < 0.05); the NIHSS score in the MDT group was lower than that in the TMC group, and the FMA score and BI score were both higher than those in the TMC group, and the difference was statistically significant (*P* < 0.05) (Figure 3).

### 4.3. Treatment Compliance

Treatment compliance was higher in the MDT group than in the TMC group, with a statistically significant difference (*P* < 0.05) (Table 2).

## 5. Secondary Complications

After care, the incidence of all types of secondary complications in Table 3 in the MDT group was less than that in the TMC group, and the difference in the incidence of shoulder subluxation, shoulder hand syndrome, and foot drop in the MDT group compared with the TMC group was statistically significant (*P* < 0.05).

## 6. Satisfaction

Patient visit satisfaction and medical staff cooperation satisfaction were both higher in the MDT group than in the TMC group, with statistically significant differences (*P* < 0.05) (Tables 4 and 5).

## 7. Discussion

AIS is the most common type of stroke in China, accounting for approximately 69.6% to 70.8% of all strokes [12]. Irreversible brain tissue damage can occur 4–6 min after the interruption of blood supply to the brain tissue in this disease, so time to resuscitation is critical to the success of treating patients with AIS [13]. The results of this study showed that the MDT group had a shorter onset—emergency physician's reception time, arrival at CT room—completion time of CT/MR, notify intervention chamber—arrival time at catheter chamber, admission—femoral artery puncture time, admission—first vessel recanalization time than the TMC group (*P* < 0.05). The reason for this is that the MDT nursing mode based on doctor-nurse-integration has optimized and improved the clinical procedures for AIS patients, such as improving the rules and regulations, clarifying the division of labor among the team members, teamwork and close cooperation, and setting time limits for each step of the process, so that each member only needs to follow the rules to achieve good results, thus gaining time for resuscitation and significantly shortening the perioperative time indicators for AIS patients. Stroke patients are prone to consciousness disorder, agitation, delirium, thinking disorder, behavior, and movement abnormalities, and the risk of unplanned extubation is high, medical personnel often take physical restraint to prevent the occurrence of unplanned extubation and other accidents, but the standardization, rationality, and effectiveness of such restraint still need to be further examined [14, 15].It is urgent to establish a standard scheme of graded physical restraint for AIS patients undergoing interventional surgery. In this result, the mean posterior constraint time of the patients in the MDT group was shorter than that of the TMC group (*P* < 0.05), suggesting that the application of MDT nursing mode based on doctor-nurse-integration can improve the accuracy of the assessment of physical constraint of stroke patients by medical staff, shorten the average body constraint time of patients, and actively promote the clinical application of standardized physical constraint management.

Previous studies [16] showed that intravascular interventional therapy with early stent removal was superior to standard medical treatment in AIS patients. The advantage of stent thrombectomy technology is that it can provide a longer treatment time window and a higher recovery rate, thus improving the clinical outcome of AIS patients [17]. In this result, the postoperative disability rate of the MDT group is lower than that of the TMC group (*P* < 0.05), suggesting that the application of the MDT nursing mode based on doctor-nurse-integration can improve the clinical outcome of AIS patients and reduce the postoperative disability rate, which is consistent with the study of Grigonyte [18]. This is mainly because the collaborative response ability of the multidisciplinary team in the MDT group can effectively shorten the treatment time window, which is very important. Emergency greenway before surgery, standardized care behaviors and resuscitation procedures during surgery, improved sickness observation and resuscitation skills of nurses, multidisciplinary assistance in timely management of postoperative complications, and timely postoperative rehabilitation guidance can improve both the efficiency of resuscitation and the prognosis of patients, thus reducing the incidence of disability. In this result, the NIHSS score of the MDT group was lower than that of the TMC group, and the FMA score and BI score were higher than those of the TMC group (*P* < 0.05), suggesting that the application of MDT nursing mode based on doctor-nurse-integration can promote the recovery of neurological and motor functions and improve the prognosis of survival quality in AIS patients after intervention surgery. The reason for this may be due to the fact that the MDT group was able to effectively shorten the time to implement various lifesaving measures during the treatment of AIS patients, and the patients were able to receive timely treatment, which facilitated the recovery of neurological and motor functions after surgery. Also, after rapid thrombectomy, the brain tissue is reperfused, which effectively reduces brain tissue damage and facilitates the recovery of neurological function, thus improving in-hospital stroke care.

The assessment of needs and potential complications associated with endovascular interventions in stroke patients in the perioperative period is essential to protect patient safety [19]. In this study, the MDT group had higher treatment compliance than the TMC group, fewer secondary complications than the TMC group, and higher patient visit satisfaction and medical staff cooperation satisfaction than the TMC group (*P* < 0.05). The reason for this is that in the care model for patients in the MDT group, the medical staff of various specialties have a reasonable division of labor, clear responsibilities, skillfull cooperation, powerful handling, and clear treatment procedures, which has promoted the improvement of teamwork among medical staff of various departments, and patients feel that there is no waiting for emergency treatment, examination, consultation, and treatment, and that various treatment measures are in place in a timely manner, which has improved patients' sense of safety and trust in the consultation, resulting in high compliance with treatment and high satisfaction with the consultation. This result is also consistent with that of He et al. [20, 21]. In addition, the MDT group's nursing measures include the implementation of perioperative health education, intraoperative optimal care, and postoperative rehabilitation guidance for patients under the integration of medical and nursing care. Through multidisciplinary collaborative consultation and nursing interventions, it not only increases the communication and exchange between doctors, nurses, and patients, but also helps anesthesiologists and surgeons to improve the efficiency of lifesaving treatment, reduces patients' negative emotions and stress reactions to fear of surgery, promotes patients' postoperative rehabilitation and enhances patients' satisfaction with their visit [22].

## 8. Conclusion

The implementation of the MDT nursing mode based on the doctor-nurse-integration for stroke patients undergoing emergency intervention surgery can improve the work efficiency of rescuing patients, improve the clinical treatment outcome of patients, and improve the satisfaction of doctors, nurses, and patients.

## Figures and Tables

**Figure 1:** Flow chart of multidepartment linkage treatment for AIS patients with emergency interventional treatment.

**Figure 2:** Perioperative time indicators. Note: (a) Onset—emergency physician's reception time (min), (b) arrival at CT room—completion time of CT/MR (min), (c) notify intervention chamber—arrival time at catheter chamber (min), (d) admission—femoral artery puncture time (min), (e) admission—first vessel recanalization time (min), (f) mean postural restraint time (h). comparison of same time indicators between groups, ^*∗*^*P* < 0.05.

**Figure 3:** Postoperative outcome indicators. Note: (a) Mortality and disability rate (%), (b) scores for each scale (scores). Comparison of same outcome indicators between groups, ^*∗*^*P* < 0.05.

**Table 1:** Baseline information.

Information	TMC group (*n* = 118)	MDT group (*n* = 87)	*t*/*χ*^2^	*P*
Age (*M* ± SD, years old)	65.14 ± 14.93	66.98 ± 11.73	0.953	0.342
Male (*n* (%))	75 (63.56)	57 (67.52)	0.084	0.772
Tobacco/alcohol history (*n* (%))	73 (61.86)	50 (57.47)	0.403	0.526
Education level (*n* (%))			1.085	0.581
Primary and below	57 (48.31)	39 (44.83)		
Secondary and below	49 (41.53)	35 (40.23)		
University and above	12 (10.16)	13 (14.94)		
Marriage status (*n* (%))			0.589	0.899
Married	93 (78.80)	72 (82.76)		
Divorced	6 (5.08)	4 (4.60)		
Widowed	13 (11.02)	8 (9.20)		
Unmarried	6 (5.08)	3 (3.44)		
Occupation (*n* (%))			1.300	0.522
On the job	12 (10.17)	11 (12.64)		
Retired	62 (52.54)	50 (57.47)		
Other	44 (37.29)	26 (29.89)		
Concomitant disease (*n* (%))			0.361	0.835
1 kind	26 (22.03)	18 (20.69)		
2 kinds	52 (44.07)	42 (48.28)		
≥3 kinds	40 (33.90)	27 (31.03)		

**Table 2:** Treatment compliance.

Grade	TMC group (*n* = 118)	MDT group (*n* = 87)	*χ * ^2^	*P*
Excellent	50 (42.37)	48 (55.17)	3.288	0.070
Good	55 (46.61)	37 (42.53)	0.337	0.561
Inferior	13 (11.02)	2 (2.30)	5.613	0.018
Excellent good rate	105 (88.98)	85 (97.70)	5.613	0.018

**Table 3:** Secondary complications.

Complication	TMC group (*n* = 118)	MDT group (*n* = 87)	*χ * ^2^	*P*
Shoulder subluxation	20 (16.95)	6 (6.90)	4.570	0.033
Shoulder hand syndrome	28 (23.73)	10 (11.49)	4.964	0.026
Foot drop	20 (16.95)	5 (5.75)	5.869	0.015
Inversion of the foot	21 (17.80)	9 (10.34)	2.226	0.136
Joint contracture	14 (11.86)	5 (5.75)	2.229	0.135
Urinary tract infection	10 (8.47)	5 (5.75)	0.549	0.459

**Table 4:** Patient visit satisfaction.

Dimension	Score range	TMC group (*n* = 118)	MDT group (*n* = 87)	*t*	*P*
Satisfaction with inpatient guidance	2∼10	7.95 ± 0.65	8.48 ± 0.70	5.584	<0.001
Satisfaction with doctors	2∼10	9.26 ± 0.72	9.68 ± 0.47	4.745	<0.001
Satisfaction with nurses	4∼20	18.14 ± 0.72	19.46 ± 0.50	14.684	<0.001
Satisfaction with doctor-nurse cooperation	4∼20	17.70 ± 0.54	19.35 ± 0.62	20.298	<0.001
Satisfaction with doctor-patient communication	6∼30	26.42 ± 1.03	28.22 ± 1.00	12.520	<0.001
Satisfaction with condition at discharge	5∼25	22.51 ± 1.02	23.53 ± 0.76	7.855	<0.001
Total satisfaction of patient visits	23∼115	102.45 ± 2.13	108.44 ± 1.74	21.471	<0.001

**Table 5:** Medical staff cooperation satisfaction.

Dimension	Score range	TMC group	MDT group	*t*	*P*
Doctor (*n* = 9)					
Doctor-nurse cooperation attitude	15∼75	58.55 ± 7.60	67.32 ± 5.51	2.803	0.013
Doctor-nurse cooperation feeling	9∼45	35.82 ± 3.22	40.87 ± 2.50	3.716	0.002
Nurse (*n* = 11)					
Doctor-nurse cooperation attitude	15∼75	61.15 ± 6.52	68.05 ± 5.54	2.675	0.015
Doctor-nurse cooperation feeling	9∼45	35.99 ± 4.40	42.36 ± 2.50	4.175	0.001

## Data Availability

The data used to support the findings of this study are available from the associated author upon reasonable request.
